# Research on the Effect of Nursing Methods for Gestational Diabetes Mellitus Based on Comprehensive Nursing Intervention

This article has been retracted.

**DOI:** 10.1155/2022/2396658

**Published:** 2022-07-14

**Authors:** Xueqiong Ren, Jianing Jin, Yaer Chen, Jing Jin

**Affiliations:** The Affiliated Hospital of Medical School of Ningbo University, Ningbo 315020, China

## Abstract

In order to explore the effective way of gestational diabetes care, this paper applies comprehensive nursing to gestational diabetes care. In terms of nursing intervention for pregnant women with gestational diabetes mellitus, combining the phased changes of pregnant women's physiological and psychological needs during pregnancy, this paper comprehensively implements health education, diet intervention, exercise intervention, pregnancy monitoring, psychological intervention, infection prevention, and perinatal monitoring and other nursing interventions in a selective and focused manner. This makes the intervention measures at each stage focused, intersecting, interpenetrating, and continuing to play a role, which can effectively improve the implementation effect of the intervention measures and better promote the effective improvement of pregnancy outcomes. In addition, this paper studies the effect of gestational diabetes care based on comprehensive nursing intervention through a controlled trial, and the study verifies that comprehensive nursing has a good effect in gestational diabetes care.

## 1. Introduction

At present, more and more studies have begun to find that if gestational diabetes patients receive correct and timely intervention during pregnancy, the prognosis of mother and baby can be significantly improved, and the incidence of complications can be significantly reduced. Moreover, a large number of studies have proved that actively cooperating with treatment is easier to control blood sugar within a satisfactory range, and effective diet and blood sugar intervention measures are the key to the treatment of gestational diabetes mellitus and the reduction of maternal and infant complications [1]. At the same time, if gestational diabetes patients are given early health education, guidance on diet, exercise, self-glucose monitoring, and insulin treatment to improve pregnant women's awareness of the disease, it can encourage patients to actively cooperate with treatment and significantly improve pregnancy outcomes. Gestational diabetes is more harmful to pregnant women and perinatal infants and will seriously affect the life safety of pregnant women and perinatal infants. In addition, the prepregnancy weight of pregnant women and the increase of weight during pregnancy have a great relationship with the occurrence of gestational diabetes mellitus. If the disease is not treated in time, it can lead to adverse pregnancy outcomes [2]. Therefore, early intervention and scientific management of gestational diabetes mellitus can reduce the perinatal morbidity. The main effects of the disease on the perinatal period include gestational hypertension, infection, polyhydramnios, macrosomia, fetal dysplasia, stillbirth, neonatal hypoglycemia, and neonatal respiratory distress syndrome. In addition, a number of studies have shown [3] that if gestational diabetes mellitus patients are diagnosed and treated promptly and correctly during pregnancy, the prognosis of mother and baby will be significantly improved, and the incidence of serious complications can be significantly reduced. Literature [4] has shown that timely and effective intervention and treatment for pregnant women with gestational diabetes can reduce the incidence of maternal and infant complications. Moreover, it is of great significance for improving the systematic management of pregnant and lying-in women, improving the quality of obstetric prevention and treatment, and reducing the “three rates,” namely, maternal mortality, perinatal mortality, and birth rate of sick and disabled children. Early intervention in pregnant women with gestational diabetes mellitus to control blood sugar within a satisfactory range is the key to improving pregnancy outcomes. Literature [5] also showed that the probability of early and midterm nursing intervention to control blood sugar at normal levels was 86.8% and 84.1%, respectively, and that of late intervention was 42.1%. It can be seen that the treatment of gestational diabetes should be detected and treated early in order to minimize the adverse effects on pregnant women, fetuses, and newborns.

With the increasing awareness of gestational diabetes, pregnant women generally attach great importance to the changes in their bodies during pregnancy, which lays a good foundation for strengthening nursing interventions during pregnancy. How to control and manage the amniotic fluid index, body weight, blood sugar, and other indicators during pregnancy is of great significance to ensure the health of mothers and babies. Some studies believe that after gestational diabetes is diagnosed, timely health education interventions will lay the foundation for the implementation of other interventions in the later stages of pregnant women with gestational diabetes [6]. Health education during pregnancy can help pregnant women and their families understand the dangers of gestational diabetes to maternal and child health, understand the common symptoms and treatment methods of gestational diabetes, and actively cooperate with various inspections, which are helpful for early detection and active cooperation. Studies have shown that the needs of gestational diabetes patients and their families for health education are urgent and multifaceted [7]. By explaining the impact of gestational diabetes on pregnant women, fetuses and newborns in simple terms, pregnant women, and their families should pay more attention to this disease. Related research believes that for gestational diabetes, health education is more important than drug treatment [8]. Research results show that implementing health education can help pregnant women with gestational diabetes to better cooperate with treatment, effectively control blood sugar, and improve pregnancy outcomes, thereby ensuring maternal and child health [9].

Health education intervention can effectively improve the diet, exercise, and personal hygiene habits of pregnant women with gestational diabetes mellitus, improve the compliance of pregnant women with gestational diabetes mellitus [10], and significantly improve pregnancy outcomes. Dietary intervention is the foundation and the most important factor in the treatment of gestational diabetes. Through dietary intervention, indicators such as weight gain during pregnancy and delivery weight can be effectively managed and controlled, thereby effectively improving pregnancy outcomes. At the same time, because dietary intervention is greatly affected by factors such as the pregnant woman herself and her family's living habits, the intervention process has many troublesome factors, and it is difficult to implement. Therefore, the simultaneous use of dietary intervention and health education and other interventions has a greater impact on improving pregnancy outcomes for a significant effect [11]. Dietary and nutritional care for gestational diabetes patients is very important. Through reasonable dietary intervention, it is beneficial to maintain the blood sugar level in a reasonable range. Dietary intervention is very necessary and very important for pregnant women with gestational diabetes mellitus. However, when implementing dietary intervention for pregnant women with gestational diabetes mellitus, the daily calorie intake should be reasonably determined based on the specific situation of each pregnant woman, while ensuring the effective supply of nutrients and heat energy for the healthy growth and development of pregnant women and their fetuses, avoiding starvation ketone bodies and postprandial hyperglycemia to occur [12]. Therefore, dietary nursing intervention plays an important role in the comprehensive nursing intervention for pregnant women with gestational diabetes mellitus. At the same time, some researchers believe that reasonable diet plus exercise therapy is the first choice for the treatment of gestational diabetes mellitus. About 75%-80% of pregnant women with gestational diabetes mellitus can adjust their blood sugar levels through lifestyle adjustments such as diet and exercise ideal range [13]. The results of the literature [14] show that nursing interventions have a positive impact on the prognosis of gestational diabetes mellitus, and its intervention effect is not inferior to the simple endocrinologist's treatment. The study of literature [15] showed that after implementing diet and exercise nursing intervention, the incidence of maternal and infant complications in the nursing intervention group was significantly lower than that in the control group in 100 pregnant women with gestational diabetes mellitus in the intervention group compared with the control group. Pregnant women with gestational diabetes have many influences and constraints during pregnancy, so a single nursing intervention is easily interfered by other factors, thus affecting the intervention effect. Judging from the current domestic and foreign research, for pregnant women with gestational diabetes mellitus, comprehensive and systematic intervention measures are more likely to produce synergistic effects and then play the best intervention effect [16].

With the rapid development of economy and society and the continuous improvement of medical level, people's attention to health and material level has also increased rapidly [17]. Pregnant women with gestational diabetes and their families pay more and more attention to the quality of pregnant women during pregnancy, and health education plays an important role in hospital management. It has been fully implemented, and dietary intervention has become a commonly accepted nursing intervention for most pregnant women, and exercise therapy is more likely to be adopted by pregnant women [18]. Nursing interventions such as psychological intervention, monitoring during pregnancy, and infection prevention are gradually being effectively applied in most studies [19]. The effect of exercise therapy for gestational diabetes patients cannot be ignored. Pregnant women with gestational diabetes maintain proper exercise, which is not only beneficial to the health of mothers and babies, but also to better control of blood sugar levels, because the exercise of but also help to improve the sensitivity of insulin and gender receptor binding [20]. Improving glucose tolerance and reducing insulin requirements in patients with gestational diabetes can be achieved through appropriate exercise. Studies have shown that exercise has a positive effect on enhancing the sensitivity of peripheral tissues to insulin, improving the uptake and utilization of glucose by muscle cells, and eliminating insulin resistance. Upper extremity exercise intervention can help improve the pregnancy outcomes of pregnant women with high risk factors for diabetes [21]. Safe and effective exercise can help rationally control the blood sugar level of pregnant women with gestational diabetes. However, the specific exercise method and single exercise time need to be combined. Each pregnant woman's own conditions are specifically determined.

Prevention is the main strategy for disease control. The realization of early prevention and control of GDM will effectively delay or avoid the occurrence of GDM, improve maternal and infant outcomes, and reduce social burden. In the research on GDM intervention, both foreign and domestic, most of them implement comprehensive nursing measures such as health education, diet, and exercise intervention, mainly through knowledge lectures, outpatient consultation, telephone follow-up, etc. After a period of follow-up, the intervention of the effect is analyzed. Most of these studies focus on groups with GDM, lack of early intervention for high-risk groups of GDM, and the intervention measures are mostly formed on the basis of previous summary, and the measures lack evidence-based support. Effective intervention needs to be based on the corresponding theory. The previous research lacks an effective theoretical basis for the discussion of why the intervention, why the individual changes, how the intervention can improve the individual's cognition, and how to ensure the compliance and continuity of the intervention.

Pregnancy is a special physiological stage for women. Patients with gestational diabetes will have a series of physiological pressures and pathogenic anxiety. If diabetes during pregnancy is not paid enough attention or treated in time, it will often bring adverse consequences to mothers and babies. To establish a harmonious and effective relative network, family members must create a good family atmosphere, be good at understanding the psychological activities of patients, patiently listen to the requirements or questions raised by patients, and provide targeted explanations and guidance, so that patients can get the system of family, friends, and medical staff. Support and timely eliminate the doubts in the heart, so as to relieve the negative emotions such as tension and fear to achieve the purpose of reducing clinical medication.

In order to improve the nursing effect of gestational diabetes mellitus, this paper applies comprehensive nursing to gestational diabetes mellitus nursing, explores the effect of comprehensive nursing, and effectively improves the nursing effect of gestational diabetes mellitus.

## 2. Materials and Methods

In this study, patients diagnosed with gestational diabetes mellitus by glucose screening in the outpatient department of obstetrics and gynecology of the hospital were selected as samples. The appropriate pregnant women who voluntarily received comprehensive nursing intervention were selected as the experimental group. The remaining gestational diabetes patients who did not receive comprehensive nursing intervention or were unwilling to receive comprehensive nursing intervention served as the control group. The relevant study design was approved by the ethics committee. Inclusion criteria are as follows: control group: pregnant women with gestational diabetes mellitus who were diagnosed with gestational diabetes mellitus in the obstetrics and gynecology outpatient clinic of the hospital according to gestational age and parity and were hospitalized in the obstetrics and gynecology department. Moreover, they did not receive or were reluctant to undertake comprehensive nursing interventions. Experimental group: the research subjects were pregnant women who underwent glucose screening in the outpatient department of obstetrics and gynecology of the hospital for less than 28 weeks of gestation and were diagnosed with gestational diabetes mellitus. Before this pregnancy, there was no threatened miscarriage, threatened premature birth, heart disease, hypertension, placenta previa, intrauterine growth retardation, etc. Those with education level above junior high school voluntarily accept comprehensive nursing intervention. The diagnostic criteria of the two groups of pregnant women were in line with the diagnostic criteria of gestational diabetes mellitus in the seventh edition of the Obstetrics and Gynecology Textbook of the People's Medical Publishing House. Exclusion criteria are as follows: pregnant women with gestational diabetes mellitus who failed to complete comprehensive nursing interventions such as health education, diet intervention, exercise intervention, and perinatal monitoring.

Comprehensive nursing intervention measures were taken for pregnant women with gestational diabetes mellitus included in the experimental group, and the implementation of intervention measures was divided into three stages. The first stage is when the gestational age is less than 28 weeks, and the experiment focused on health education, supplemented by diet control and exercise intervention. The second stage is from 28 to 36 gestational weeks. The experiment focused on diet intervention, exercise intervention, pregnancy care and self-monitoring, and health education and psychological counseling for pregnant women. The third stage is from 36 gestational weeks to postpartum. While focusing on psychological intervention, infection prevention, and perinatal monitoring, the experiment continued to carry out health education, dietary control, and maternal blood glucose monitoring. The intervention measures in the above three stages are focused on, intersect, penetrate each other, and continue to play a role in different stages. During the nursing intervention process, the pregnant women should be followed up every two weeks for dietary intervention, exercise intervention, nursing during pregnancy, self-monitoring, and blood sugar control. At the same time, it is necessary to communicate and solve new problems with pregnant women in a timely manner, so as to improve the compliance of pregnant women with nursing intervention, in order to achieve the best nursing intervention effect. Blood sugar control standard is as follows: fasting blood sugar less than 5.3 mmol/L, 2 hours postprandial blood sugar less than 6.7 mmol/L. Pregnant women and newborns with gestational diabetes mellitus included in the control group were treated with traditional nursing methods. By comparing the differences in maternal and infant outcomes between the experimental group and the control group, the effect of comprehensive nursing intervention on the pregnancy outcomes of the most gestational diabetes mellitus was systematically reviewed.

During pregnancy, pregnant women with gestational diabetes are prone to a series of special changes in physiology and psychology due to lack of effective understanding of pregnancy and fear of gestational diabetes, resulting in elevated blood sugar, which threatens and affects the health of mothers and babies. Therefore, timely health education intervention can enable pregnant women to have a comprehensive understanding of pregnancy and diabetes and improve the compliance of pregnant women and their families with dietary intervention and exercise intervention. Furthermore, it helps to adjust and improve the pregnancy environment of pregnant women with gestational diabetes mellitus and helps to promote good outcomes for mothers and infants. In the early stage of health education intervention in this study, a professional gestational diabetes health education group was established, which consisted of senior obstetrics and gynecology experts, obstetric nurses, endocrinology experts, and nutritionists. For the gestational diabetes patients and their families in the experimental group, we formulated a targeted health education intervention plan based on the actual situation of each pregnant woman. In addition, the experiment carried out publicity and education on gestational diabetes related knowledge through multimedia teaching, mobile phone text messages, establishment of WeChat, groups, health education video clips, and bedside one-on-one. At the same time, we introduced knowledge about gestational diabetes to patients, so that they can understand that appropriate scientific intervention can greatly improve adverse pregnancy outcomes, so as to ensure good compliance among educated people. In addition, we guided pregnant women to understand the disease comprehensively, objectively, and correctly, improve the negative emotions of pregnant women with gestational diabetes mellitus, maintain a good and stable psychological state, and promote smooth and healthy childbirth. In addition, we organize and carry out collective psychological counseling, give full play to the role of collective education, and organize pregnant women in the experimental group to participate in weekly knowledge counseling and expert lectures for gestational diabetes patients. Further, we try to guide the group to create a good atmosphere and psychological orientation of optimism and face up to reality, to encourage them to support and encourage each other, and to ensure that the interventions of diet and exercise are put into place. According to the specific conditions of each pregnant woman in the experimental group, such as blood sugar level and body mass index, a personalized dietary intervention plan was reasonably determined to ensure the effective supply of nutrients needed by pregnant women during pregnancy and healthy growth and development of the fetus. We educated pregnant women with gestational diabetes mellitus in the experimental group to combine their own physical conditions with appropriate exercise. At the same time, we educated them to pay close attention to their own feelings, scientifically grasp the time and intensity of each exercise, ensure that the exercise is safe, effective, and reasonable, and avoid exercising on an empty stomach as much as possible. Moreover, we instructed pregnant women with gestational diabetes mellitus in the experimental group to master their own methods of checking blood sugar and make records. In addition, we educate and guide pregnant women with gestational diabetes mellitus, adhere to regular weight measurement, master weight changes, adhere to regular daily blood pressure measurement, observe blood pressure fluctuations, and make relevant records carefully. After the gestational age reached 28 weeks, we taught the pregnant women in the experimental group how to count fetal movements and record them. If there is a decrease in fetal movement, the number of fetal movements per hour is less than 4 times, or the fetal movement is too frequent, and the number of fetal movements per 12 hours exceeds 40 times; the pregnant woman should go to the hospital for examination and treatment in time accompanied by her family to effectively rule out intrauterine distress. In addition, we instructed the pregnant women in the experimental group to develop good hygiene habits, pay attention to indoor hygiene, change and wash intimate clothing every day, especially pay attention to strengthening personal oral hygiene, and pay attention to maintaining perineal hygiene to effectively enhance their own resistance. If pregnant women find symptoms of infection during pregnancy, they should contact the competent doctor in time and take effective treatment measures in time, so that the symptoms of infection can be effectively controlled in time to avoid the expansion of infection.

In the second and later stages of pregnancy, through the intervention of health education in the previous stage, pregnant women have a certain understanding of pregnancy and diabetes. On this basis, combined with the staged needs of pregnant women and fetuses for healthy development, dietary intervention, exercise intervention, and pregnancy monitoring were implemented. At the same time, health education interventions need to continue to be carried out to ensure the effective implementation of dietary interventions, exercise interventions, and pregnancy monitoring. Through a full range of comprehensive nursing interventions, pregnant women are guided to achieve good physical and psychological outcomes.

## 3. Result

The amniotic fluid index, BMI, weight gain during pregnancy, delivery weight, fasting blood sugar, and 2 h postprandial blood sugar in the experimental group of pregnant women with gestational diabetes are lower/lower than those in the control group. The results of statistical analysis show that the differences between the experimental group and the control group in the above indicators are statistically significant (*P* < 0.05), as shown in Tables 1–6, and the corresponding statistical graphs are shown in Figures 1–6.

## 4. Analysis and Discussion

The comparison of pregnancy outcome indicators between the experimental group and the control group shows that there are no cases of gestational hypertension in the experimental group, while many cases of gestational hypertension occurred in the control group. The comparison of pregnancy outcome indicators between the experimental group and the control group shows that there are no cases of gestational hypertension in the experimental group, while many cases of gestational hypertension occurred in the control group. There is statistically significant difference in the incidence of gestational hypertension between the two groups (*P* < 0.05). Regarding the preterm birth index, the preterm birth rate of the experimental group and the control group in the control group is higher than that in the experimental group, and the statistical analysis showed that the difference is statistically significant (*P* < 0.05). The comparison result of the cesarean section rate shows that the control group was higher than the experimental group, and the statistical analysis showed that the difference is statistically significant (*P* < 0.05).

The comparison of the incidence of polyhydramnios shows that the control group was higher than the experimental group, and the statistical analysis shows that the difference was statistically significant (*P* < 0.05). The comparison results of fetal distress rate show that the real control group was higher than the experimental group, and the statistical analysis shows that the difference was statistically significant (*P* < 0.05). The comparison of postpartum hemorrhage rate shows that the control group is higher than the experimental group, and the statistical analysis shows that the difference is statistically significant (*P* < 0.05). The comparison of urinary system infection rate shows that the control group is higher than the experimental group, and the statistical analysis showed that the difference is statistically significant (*P* < 0.05). There is no significant difference in the incidence of placenta previa and premature rupture of membranes between the experimental group and the control group (*P* < 0.05). In conclusion, in addition to placenta previa and premature rupture of membranes, in the comparison of pregnancy outcome indicators such as gestational hypertension, premature birth, cesarean section, polyhydramnios, fetal distress, postpartum hemorrhage, and urinary tract infection, the incidence rates of related pregnancy outcomes in the control group are higher than those in the experimental group, and the differences are statistically significant (*P* < 0.05).

With the increasing awareness of gestational diabetes, pregnant women generally attach great importance to the changes in their bodies during pregnancy, which lays a good foundation for strengthening nursing interventions during pregnancy. Moreover, how to control and manage the amniotic fluid index, body weight, blood sugar, and other indicators during pregnancy is of great significance to ensure the health of mothers and babies. Health education intervention can effectively improve the diet, exercise, and personal hygiene habits of pregnant women with gestational diabetes mellitus, improve the compliance of pregnant women with gestational diabetes mellitus, and significantly improve pregnancy outcomes. In addition, dietary intervention is the basis and the most important factor in the treatment of gestational diabetes. Through dietary intervention, indicators such as weight gain during pregnancy and delivery weight can be effectively managed and controlled, thereby effectively improving pregnancy outcomes. At the same time, dietary intervention is greatly affected by factors such as the pregnant woman herself and her family's living habits, and there are many troublesome factors in the intervention process, making it more difficult to implement. Therefore, the simultaneous use of dietary interventions and interventions such as health education has a more significant effect on improving pregnancy outcomes. Moreover, dietary and nutritional care of patients with gestational diabetes mellitus is very important. Through reasonable dietary intervention, it is beneficial to maintain the blood sugar level in a reasonable range, and dietary intervention is very necessary and very important for pregnant women with gestational diabetes mellitus. However, when implementing dietary intervention for pregnant women with gestational diabetes mellitus, the daily calorie intake should be reasonably determined based on the specific conditions of each pregnant woman. While ensuring the effective supply of nutrients and heat energy for the healthy growth and development of pregnant women and their fetuses, avoid starvation ketone bodies and postprandial hyperglycemia. Therefore, dietary nursing intervention plays an important role in the comprehensive nursing intervention for pregnant women with gestational diabetes mellitus.

The effect of exercise therapy for gestational diabetes patients cannot be ignored. Pregnant women with gestational diabetes maintain proper exercise, which is not only beneficial to the health of mothers and babies, but also to better control of blood sugar levels. The reason is that the movement of skeletal muscle can not only consume energy but also help to increase the sensitivity of insulin binding to receptors. Improving glucose tolerance and reducing insulin requirements in patients with gestational diabetes can be achieved through appropriate exercise. Studies have shown that exercise has a positive effect on enhancing the sensitivity of peripheral tissues to insulin, improving the uptake and utilization of glucose by muscle cells, and eliminating insulin resistance. Moreover, upper extremity exercise intervention can help improve the pregnancy outcomes of pregnant women with high risk factors for diabetes, and safe and effective appropriate exercise can help to reasonably control the blood sugar level of pregnant women with gestational diabetes. However, the specific exercise method and the single exercise time need to be determined in combination with each pregnant woman's own conditions.

## Figures and Tables

**Figure 1:** Statistical diagram of amniotic fluid index.

**Figure 2:** Statistical diagram of BMI.

**Figure 3:** Statistical diagram of weight gain during pregnancy.

**Figure 4:** Statistical diagram of weight at delivery.

**Figure 5:** Statistical diagram of fasting blood glucose.

**Figure 6:** Statistical diagram of 2 h postprandial blood glucose.

**Table 1:** Comparison table of amniotic fluid index.

Number	Test group (mm)	Control group (mm)
1	107.03	172.97
2	117.96	77.59
3	125.28	85.91
4	100.30	80.93
5	80.80	164.31
6	99.40	123.96
7	132.38	143.18
8	90.80	154.63
9	100.71	165.31
10	95.07	77.64
11	107.68	102.38
12	114.18	112.90
13	103.34	90.70
14	94.96	110.48
15	109.01	102.24
16	96.91	149.07
17	108.92	75.00
18	107.65	107.06
19	111.35	155.72
20	90.42	168.96
21	104.12	129.11
22	123.87	111.67
23	94.35	138.21
24	80.80	100.56
25	120.54	143.04
26	125.74	82.57
27	132.14	136.48
28	110.22	100.65
29	113.57	109.97
30	113.07	144.23
31	103.70	161.84
32	114.06	92.76
33	117.03	149.19
34	86.49	146.41
35	115.53	122.26
36	93.94	112.31
37	116.73	85.12
38	86.40	151.97
39	121.13	163.18
40	126.77	81.72

**Table 2:** Comparison table of BMI.

Number	Test group (kg/m^2^)	Control group (kg/m^2^)
1	18.86	18.94
2	20.31	18.05
3	21.71	17.78
4	20.21	17.62
5	19.77	22.92
6	19.74	24.54
7	20.18	20.96
8	20.91	19.28
9	19.86	20.49
10	20.06	24.36
11	20.52	17.40
12	18.84	17.50
13	20.34	18.48
14	21.51	20.26
15	20.54	24.45
16	19.62	24.18
17	20.16	17.51
18	21.15	19.37
19	20.87	20.70
20	21.65	17.59
21	19.66	23.71
22	21.94	22.96
23	19.93	18.34
24	20.13	19.30
25	21.75	18.65
26	20.31	24.05
27	20.29	21.95
28	19.43	23.32
29	21.52	20.42
30	19.42	18.62
31	20.36	23.70
32	19.27	21.47
33	21.65	24.66
34	21.22	22.20
35	19.40	24.66
36	20.17	24.42
37	20.68	19.25
38	19.64	19.60
39	20.46	19.02
40	19.18	18.09

**Table 3:** Comparison table of weight gain during pregnancy.

Number	Test group (kg)	Control group (kg)
1	18.69	20.97
2	15.98	18.64
3	15.69	16.94
4	17.37	21.65
5	15.61	16.60
6	16.68	14.86
7	17.37	19.39
8	18.37	13.99
9	15.65	17.33
10	17.18	20.54
11	15.46	16.81
12	18.15	12.69
13	19.22	16.35
14	15.53	13.68
15	17.96	21.65
16	18.15	22.28
17	15.53	18.83
18	17.53	23.24
19	15.49	12.60
20	15.73	21.94
21	17.22	22.70
22	17.93	22.35
23	18.37	23.18
24	17.12	13.36
25	18.79	22.74
26	17.96	12.63
27	19.38	18.10
28	16.11	20.88
29	17.71	22.03
30	15.73	13.84
31	16.05	16.14
32	18.76	20.91
33	15.32	16.38
34	19.31	12.44
35	17.38	14.99
36	19.27	22.00
37	17.46	13.40
38	17.32	14.14
39	15.86	13.98
40	17.04	22.12

**Table 4:** Comparison table of weight at delivery.

Number	Test group (kg)	Control group (kg)
1	68.99	70.59
2	64.77	76.99
3	64.09	62.18
4	67.84	76.46
5	62.16	68.01
6	68.15	72.15
7	73.71	73.02
8	62.39	62.25
9	72.89	78.20
10	64.04	67.86
11	73.50	74.61
12	61.66	75.61
13	64.26	61.24
14	73.78	65.98
15	64.89	69.54
16	64.34	75.81
17	62.16	66.62
18	67.23	69.21
19	62.26	79.12
20	74.48	70.56
21	74.62	68.94
22	66.68	62.07
23	62.56	79.27
24	68.67	67.18
25	63.42	62.55
26	64.98	67.50
27	67.93	73.76
28	74.35	65.81
29	61.29	74.25
30	74.73	77.00
31	72.70	63.62
32	73.28	71.97
33	74.04	68.85
34	66.15	69.77
35	63.39	66.84
36	72.13	64.00
37	65.93	65.78
38	68.30	74.39
39	61.31	66.17
40	73.50	67.24

**Table 5:** Comparison table of fasting blood glucose.

Number	Test group (mmol/L)	Control group (mmol/L)
1	4.48	5.49
2	4.59	6.09
3	5.32	6.09
4	4.26	5.93
5	4.68	5.40
6	4.43	6.12
7	4.77	5.29
8	5.29	5.24
9	4.41	5.37
10	5.23	4.98
11	4.13	6.08
12	5.10	4.90
13	5.30	5.82
14	3.97	5.23
15	4.81	5.75
16	4.36	5.67
17	4.89	5.78
18	4.50	5.65
19	5.02	5.95
20	4.08	5.66
21	5.07	5.38
22	4.68	5.59
23	4.71	5.90
24	4.52	4.70
25	5.09	5.37
26	4.95	6.17
27	5.31	5.72
28	4.88	5.32
29	4.64	5.81
30	5.24	5.92
31	4.24	5.84
32	5.06	5.46
33	4.36	5.31
34	5.08	4.80
35	4.82	5.30
36	4.02	4.86
37	4.13	4.79
38	5.20	4.97
39	4.65	5.43
40	5.26	4.74

**Table 6:** The comparison table of 2 h postprandial blood glucose.

Number	Test group (mmol/L)	Control group (mmol/L)
1	6.17	6.55
2	6.52	6.72
3	6.43	7.59
4	6.87	6.32
5	5.96	6.35
6	5.92	6.65
7	6.29	6.38
8	6.61	6.92
9	6.19	7.35
10	5.89	6.21
11	6.57	5.99
12	6.54	5.93
13	5.49	6.93
14	6.55	6.46
15	5.58	6.35
16	5.56	6.38
17	5.98	6.93
18	6.48	6.84
19	6.19	6.35
20	5.90	6.38
21	5.30	6.34
22	6.85	6.94
23	6.54	6.48
24	6.35	6.86
25	5.47	6.32
26	6.25	6.58
27	6.34	6.45
28	5.37	6.67
29	5.96	6.38
30	6.41	7.91
31	5.99	10.28
32	5.91	6.92
33	5.52	6.32
34	5.92	11.07
35	6.21	7.41
36	6.10	6.35
37	6.21	6.84
38	5.79	6.35
39	5.56	6.38
40	5.40	6.67

## Data Availability

The labeled dataset used to support the findings of this study are available from the corresponding author upon request.
